# Analysis of the Influence of Serum MMP-2 and vWF Levels on the Predictive Value of Risk Grade and Prognosis of Patients with Acute Myeloid Leukemia

**DOI:** 10.1155/2022/1865189

**Published:** 2022-07-19

**Authors:** Min Liu, Qi Yang, Licui Zhang

**Affiliations:** ^1^Department of Reproductive Medicine, First Affiliated Hospital, School of Medicine, Shihezi University, Shihezi, Xinjiang 832003, China; ^2^Clinical Laboratory, First Affiliated Hospital, School of Medicine, Shihezi University, Shihezi, Xinjiang 832003, China

## Abstract

The expression of serum MMP-2 and von Willebrand factor (vWF) in patients with acute myeloid leukemia (AML) at different risks and their predictive value and prognostic impact were investigated. A total of 105 AML patients admitted to our hospital from February 2020 to February 2022 are divided into group A (32 cases), group B (46 cases), and group C (27 cases) according to risk stratification from low to high. The patients in the three groups are treated with induction chemotherapy according to the risk grade, and the expression of serum matrix metalloproteinase-2 (MMP-2) and vWF antigen in the three groups are detected before and after treatment. Pearson correlation is used to analyze the correlation between MMP-2 and vWF expression and prognosis of AML patients. ROC curve is used to analyze the predictive value of MMP-2 and vWF expression for risk grading of AML patients. MMP-2 and vWF are highly expressed in middle and high-risk patients, had high predictive value for the risk grade of AML patients, and are correlated with the prognosis of AML patients to a certain extent.

## 1. Introduction

Acute myelocytic leukemia (AML) is a hematologic malignant tumor, which is mainly caused by the malignant transformation of hematopoietic progenitor cells. AML can invade various organs such as the liver, spleen, and lymph nodes, threatening people's life safety [1, 2]. The acute leukemia incidence of AML is at higher levels, about 1.62/10 [3], and still has the growth of the clinical manifestation of bleeding, infection, and symptoms such as abnormal temperature rise and the body metabolic disorder, and due to the nature of the cells in patients with drug resistance increased and reduced sensitivity to drugs, only 20% of the patients can be fully cured; these diseases have a high recurrence rate [4, 5], and these diseases are characterized by acute onset. The risk level of newly diagnosed cases is mostly medium-risk type. At present, clinical tests are mostly carried out based on cytogenetics and other indicators, and the auxiliary judgment of multiple examinations is required, and the detection methods are complicated [6].

In order to improve the treatment level of patients with different risk grades of AML and improve the prognosis of patients, effective biological markers should be sought to improve the prediction level of risk grades. Matrix metalloproteinase-2 (MMP-2) is a cellular hydrolytic enzyme that can degrade extracellular matrix and participate in physiological processes such as cell differentiation and migration. It can promote the metastasis of tumor cells by destroying the matrix membrane and play an important role in the generation and development of tumors. It has a certain correlation with the prognosis of tumor patients and has been used as a marker of tumor detection and prognosis in various cancer studies [7]. vWF can reflect the hypercoagulability of blood and the damage of vascular endothelial cells and is an effective indicator for the risk classification of AML patients [8]. To improve the prediction level of AML risk grade and prognosis, this study analyzed the expression of MMP-2 index and vWF antigen in patients with different AML risk grades and the correlation between the two indexes and prognosis, in order to provide a reference value for clinical practice.

The rest of this study is organized as follows: Section 2 discusses related work, followed by data information and treatment methods designed in Section 3.  Section 4 shows the experimental results, and Section 5 concludes the study with summary and future research directions.

## 2. Related Work

Risk stratification treatment for patients with AML is according to the different degrees of disease for the appropriate treatment, including the selection of drug dosage, the strength, and degree of drug resistance in patients with chemotherapy, is from the largest extent, and can reduce the different intensities of chemotherapy in patients with low, medium, and high kinds of dangerous level which have an adverse effect on body and curative effect [9, 10]. AML is a high incidence type of acute leukemia, and the essence of its pathogenesis is the malignant proliferation of leukemia cells in bone marrow, resulting in the accumulation of a large number of myeloid precursor cells in bone marrow, and hematopoietic disorder is due to abnormal proliferation and blocked apoptosis of hematopoietic cells [11, 12]. The mechanism of MMP-2 in AML patients is that it can hydrolyze the stromal membrane of tumor cells, enhance the adhesion between cells, and provide important conditions for the proliferation of tumor cells. Meanwhile, tumor cells can also stimulate the body to produce a large amount of MMP-2, which plays an important role in their own growth and migration [13]. vWF is a polymeric glycoprotein synthesized by megakaryocytes and vascular endothelial cells. When vascular endothelial cells are damaged, a large number of vWF will be detected in plasma, and platelets will accumulate on the surface of thrombus, resulting in hypercoagulability of blood, resulting in hematopoietic dysfunction in AML patients, thrombosis, and other complications [14, 15]. Research by Saleh et al. [16] showed that MMP-2 high expression can interact with multiple inflammatory factors in vivo, participate in the infiltration and metastasis of tumor cells, and accumulate in large numbers in high-risk patients.

The results of research are consistent with the conclusion that MMP-2 index increased with the increase of risk coefficient, which may be due to the fact that MMP-2 has the important function of decomposing matrix membrane, which can regulate the growth of tumor cells. Matrix membrane is a basement membrane that AML cells must pass through to enter blood cycle. High expression of MMP-2 predicts the risk of continuous growth, invasion, and metastasis of AML patients, according to the results of this study of three groups of patients after treatment vWF antigen levels are reduced, but the vWF antigen levels and the incidence of complications with increasing risk classification and corresponding increase, the reason may be due to the high degree of high-risk patients with tumor progression, and AML cells stimulate vascular endothelial cells release a lot of vWF and make high blood coagulation state. At the same time, it has become a risk factor for inducing venous thrombosis complications in patients, which is consistent with the research results of relevant scholars [17–19].

In addition, MMP-2 and vWF indexes showed a positive trend of change with the increase of the incidence of complications, suggesting a certain influence on the prognosis of AML patients with different risk grades. Analysis of the reason for their existence is that AML cells can produce a variety of decomposition enzymes such as MMP-2 and MMP-9, which can promote cell invasion and metastasis. Low expression of MMP-2 in patients with different grades indicates remission of AML patients, reduced differentiation of tumor cells, and fewer complications. Therefore, low expression of MMP-2 may indicate a good prognosis [20, 21]. The decrease of vWF antigen content in AML patients indicates the presence of a small amount of vascular endothelial cell activation and thrombosis or the absence of thrombosis and also indicates the reduction of AML stimulation to AML patients. Therefore, the decrease of vWF content detected in plasma has a good indication of prognosis. The results of this study showed that the expression of MMP-2 and vWF indicators had certain predictive value for the risk grade of AML patients, indicating that the higher the risk degree of AML, the level of MMP-2 index in vivo also is increased, and the MMP-2 index showed high expression, and the vWF content is higher abnormally. The analysis reason is that when AML patients are in different grades, the growth and invasion degree of AML malignant cells in vivo are different, and the higher the risk degree, the higher the differentiation degree of AML malignant cells and the higher the damage degree of vascular endothelial cells, thus the high expression of vWF [22, 23].

## 3. Data Information and Treatment Methods

### 3.1. General Information

A total of 105 AML patients admitted to our hospital from February 2020 to February 2022 are divided into three groups according to their cytogenetic and molecular biological detection indexes at admission. The risk stratification is from low to high, respectively, A–C groups. There are 32 patients in group A, including 16 males and 16 females. The average age is (45.26 ± 6.02) years from 36 to 66 years. The cell content of bone marrow is (41.52 ± 5.11) %. Group B (46 cases) includes 24 males and 22 females. The average age is (43.41 ± 7.21) years from 37 to 61 years. The cell content of bone marrow is (43.52 ± 6.01) %. Group C (27 cases) includes 14 males and 13 females. The average age is (42.76 ± 8.02) years from 35 to 65 years. The content of bone marrow cells is (43.52 ± 6.35) %, and there is no significant difference in general data among all groups (*P* > 0.05). All patients participating in the study understood the content and purpose of the study in detail and obtained consent from patients and signed informed consent.

### 3.2. Treatment Methods

#### 3.2.1. Treatment Methods

The three groups received induction chemotherapy as follows: groups A and B received low-intensity induction chemotherapy, mitoxantrone 4 mg·m^−2^·d^−1^ × 3 d for 3 consecutive days, hartaxoline 1.25 mg·m^−2^·d^−1^, and cytarabine 50 mg·m^−2^·d^−1^. Group C received mitoxantrone 8 mg·m^−2^·d^−1^, hartonine 2.5 mg·m^−2^·d^−1^, and cytarabine 50 mg·m^−2^·d^−1^.

#### 3.2.2. Determination of Matrix Metalloproteinase-2 (MMP-2) in Serum

In the morning, 3 ml of venous blood is extracted from the patients in the three groups on an empty stomach. Centrifuge (5910R, Ebender, Germany) is centrifuged at a speed of 2500 r/min for 15 min for centrifugation, and the supernatant is stored in a refrigerator at −80°C. Detection method: the double antibody one-step Sandwich method, ELISA kit (JLC-G3760, Shanghai Ren Jie Biotechnology Co., LTD.) is used to add specimens, standard materials, and HRP labeled detection antibodies into the coated micropores of human captured antibodies in advance. After incubation and thorough washing, TMB color is displayed. Measure the absorbance (OD value) at 450 nm with a microplate meter and calculate the blank value after reducing all OD values. Standard 20, 10, 5, 2.5, 1.25, 0.625, 0.312, and 0 ng/ml are taken as abscissa and OD value as ordinate, plot on coordinate paper, and draw the standard curve. The corresponding MMP-2 content is found on the curve according to the sample OD value.

#### 3.2.3. Plasma von Willebrand Factor (vWF) Antigen Detection

The detection procedures of the human plasma vWF antigen detection kit (ZY-VWF-HU, Shanghai Zeye Biotechnology Co., Ltd.) are as follows: take out the required strips and set the standard and sample wells, add standard 50 *μ*L of different concentrations to each standard well, and add test sample 50 *μ*L to blank well. In addition to blank wells, horseradish peroxidase (HRP) labeled detection antibody 100 is added to each well of standard and sample wells. The reaction wells are sealed with elbow plate membrane and incubated for 60 min in a 37°C waterbath or thermostat. Dry on washcloth, add washing solution (350 *μ*L) to each well, and let stand for 1 min. Discard washing liquid, pat dry on absorbent paper, and repeat washing plate 5 times. Add substrate A and substrate B 50 *μ*L to each well and incubate at 37°C for 15 min away from light. Add stop solution 50 *μ*L to each well and measure the OD value of each well at 450 nm within 15 min. The standard curve is drawn with the logarithm of dilution of normal mixed plasma as abscissa and the corresponding optical density value as ordinate. The vWF level of mixed plasma is set at 100%. The measured optical density value of samples is substituted into the standard curve to obtain the amount of vWF antigen in the samples (%).

### 3.3. Statistical Treatment

Statistical data are processed by SPSS 24.0 software, measurement data are expressed as (‾*x* ± *s*), intergroup data are tested by the *t*-test, multigroup data are tested by the F test, and count data are expressed by the *χ*^2^ test, %. Pearson coefficient is used for correlation analysis. ROC curve is used to analyze the predictive value of MMP-2 and vWF expression on the risk grade of AML patients. When *P* < 0.05, the difference between data is considered statistically significant.

## 4. Experimental Results

### 4.1. Comparison of Serum MMP-2 Expression before and after Treatment among the Three Groups

Table 1 provides the change in the expression levels of MMP-2 in the three groups (‾*x* ± *s*, ng/mL). In Table 1, a and b, respectively, represent a comparison of group A and group B, *P* < 0.05.  Figure 1 shows the serum MMP-2 expression levels of the three groups at different time points. It is evident from Table 1 and Figure 1 that the MMP-2 level of group C is higher than that of group A and group B at two time points before and after treatment, and group B is higher than that of group A. After treatment, the MMP-2 level of the three groups shows that A has a decreasing trend, and the data show statistical differences (*P* < 0.05).

### 4.2. Comparison of vWF Antigen Content between the Three Groups before and after Treatment

Table 2 provides the vWF level changes in the three groups. In Table 2, a and b, respectively, represent a comparison of group A and group B, *P* < 0.05.  Figure 2 shows the serum vWF expression levels of the three groups at different time points. It is evident from Table 2 and Figure 2 that the vWF level of group C is higher than that of group A and group B at two time points before and after treatment, and group B is higher than that of group A. After treatment, the vWF level of the three groups shows A decreasing trend, and the data show statistical differences (*P* < 0.05).

### 4.3. Comparison of the Incidence of Complications among the Three Groups within One Year after Follow-Up Treatment

Table 3 provides the difference in the complication rate of the three groups. In Table 3, a and b, respectively, represent a comparison of group A and group B, *P* < 0.05. It is evident from Table 3 that group C has a higher proportion of complications than groups A and B, and the proportion of group B is higher than group A, with statistical differences (*P* < 0.05).

### 4.4. Correlation Analysis of MMP-2 and vWF Expression and Prognosis of AML Patients

Table 4 provides the correlation analysis of MMP-2 and vWF expression with a prognosis of AML patients. It is evident from Table 4 that MMP-2 expression and vWF antigen content are positively correlated with the incidence of complications (*P* < 0.05).

### 4.5. Predictive Value of MMP-2 and vWF Expression for Risk Grading of AML Patients

Table 5 provides the predictive value of MMP-2 and vWF expression for risk grading of AML patients.  Figure 3 shows the ROC curve of the predictive value of MMP-2 and vWF expression for risk grading of AML patients. It is evident from Table 4 and Figure 3 that the predictive value of MMP-2 and vWF expression on the risk grading of AML patients is higher under the ROC curve, and MMP-2 is higher than vWF. Both indicators had high specificity and sensitivity.

## 5. Conclusion and Future Work

Although this study has achieved certain results, there is less sample size, for the time limit index selection is not the problem, and some deficiencies still exist in research; in the subsequent scholars' study, can enrich study sample size and selection of several indicators to make the research achievements of different dangerous degree classification of AML patients more comprehensive and scientific.

Above all, MMP-2 and vWF indicators in different dangerous degree classifications have different expressions in patients with AML and in the dangerous degree have high expression in a high degree of risk; the risk classification of patients with AML has higher predictive value and positively related with the complications in patients with AML, and its prognosis has certain implications.

## Figures and Tables

**Figure 1:** Serum MMP-2 expression levels of the three groups at different time points.

**Figure 2:** Serum vWF expression levels of the three groups at different time points.

**Figure 3:** ROC curve of the predictive value of MMP-2 and vWF expression for risk grading of AML patients.

**Table 1:** The change in the expression levels of MMP-2 in the three groups (‾*x* ± *s*, ng/mL).

Group	Pretherapy	Posttreatment
A group (*n* = 32)	413.45 ± 59.23	211.56 ± 41.22
B group (*n* = 46)	431.55 ± 65.41^a^	232.44 ± 53.41^a^
C group (*n* = 27)	463.36 ± 54.32^ab^	255.43 ± 47.63^ab^
*F*	21.231	20.143
*P*	<0.001	<0.001

**Table 2:** vWF level changes in the three groups (‾*x* ± *s*, %).

Group	Pretherapy	Posttreatment
A group (*n* = 32)	213.14 ± 109.23	174.23 ± 98.42
B group (*n* = 46)	231.55 ± 114.31^a^	193.23 ± 86.23^a^
C group (*n* = 27)	263.29 ± 100.32^ab^	220.65 ± 96.44^ab^
*F*	20.131	21.112
*P*	<0.001	<0.001

**Table 3:** The difference in the complication rate of the three groups (*n*, %).

Group	Infectious lesions (%)	Venous thrombus (%)	Intracranial tumor (%)	Overall incidence (%)
A group (*n* = 32)	9 (28.13)	9 (28.13)	0 (0.00)	18 (56.25)
B group (*n* = 46)	16 (34.78)	12 (26.09)	1 (2.17)	29 (63.04)^a^
C group (*n* = 27)	10 (37.04)	13 (48.15)	2 (7.41)	24 (88.89)^ab^
*x* ^2^	20.131	21.142	22.369	23.411
*P*	0.002	<0.001	<0.001	<0.001

**Table 4:** Correlation analysis of MMP-2 and vWF expression with a prognosis of AML patients.

Metric infectious lesion (%)	MMP-2		vWF	
	*r*	*P*	*r*	*P*
Venous thrombus (%)	0.604	0.007	0.562	0.008
Intracranial tumor (%)	0.565	0.008	0.607	0.006
Metric	0.587	0.005	0.684	0.004

**Table 5:** Predictive value of MMP-2 and vWF expression for risk grading of AML patients.

Index	Sensitivity	Specificity	AUC	95% CI	Youden index
MMP-2	81.50	62.05	0.785	0.627–1.011	0.434
vWF	75.55	60.05	0.755	0.655–0.944	0.356

## Data Availability

The data used to support the findings of this study are available from the corresponding author upon request.
